# Alzheimer's Disease Prediction Algorithm Based on Group Convolution and a Joint Loss Function

**DOI:** 10.1155/2022/1854718

**Published:** 2022-10-12

**Authors:** Jiayuan Cheng, Huabin Wang, Shicheng Wei, Fei Liu, Yonglin Chen

**Affiliations:** ^1^International Brain Science and Engineering Center, School of Computer Science and Technology, Anhui University, Hefei 230039, China; ^2^School of Electrical and Information Engineering, University of Sydney, Sydney 2006, Australia

## Abstract

Alzheimer's disease (AD) can effectively predict by 18F-fluorodeoxyglucose positron emission tomography (18F-FDG PET) of the brain, but current PET images still suffer from indistinct lesion features, low signal-to-noise ratios, and severe artefacts, resulting in poor prediction accuracy for patients with mild cognitive impairment (MCI) and unclear lesion features. In this paper, an AD prediction algorithm based on group convolution and a joint loss function is proposed. First, a group convolutional backbone network based on ResNet18 is designed to extract lesion features from multiple channels, which makes the expression ability of the network improved to a great extent. Then, a hybrid attention mechanism is presented, which enables the network to focus on target regions and learn feature weights, so as to enhance the network's learning ability of the lesion regions that are relevant to disease diagnosis. Finally, a joint loss function, that avoids the overfitting phenomenon, increases the generalization of the model, and improves prediction accuracy by adding a regularization loss function to the conventional cross-entropy function, is proposed. Experiments conducted on the public Alzheimer's Disease Neuroimaging Initiative (ADNI) dataset show that the algorithm we proposed gives a prediction accuracy improvement of 2.4% over that of the current AD prediction algorithm, thus proving the effectiveness and availability of the new algorithm.

## 1. Introduction

Alzheimer's disease (AD) is a kind of clinical neurodegenerative disease. Short-term memory loss is an early symptom of the condition, as the disease progresses, patients may develop language impairment, disorientation, and many behavioural problems. Eventually, the patient loses physical function, which leads to death. There is still no effective treatment to stop or reverse the progression of the disease [1].

To assist in the diagnosis of AD, clinicians utilize positron emission tomography (PET), magnetic resonance imaging (MRI), medical imaging techniques such as computed tomography (CT), and other techniques. Among them, PET can image the metabolic and functional statuses of brain lesion regions. Due to this property, PET-based neuroimaging diagnosis is an important method for the diagnosis of AD in the early stage. If patients with mild cognitive impairment (MCI), a state between AD and normal control (NC), can be screened early and treated, further deterioration of the disease can be delayed.

Recently, the achievements of Convolutional Neural Network (CNN) in the diagnosis of brain diseases are increasingly recognized [2]. Syaifullah et al. [3] combined a voxel-based morphometry (VBM) with support vector machine (SVM) to construct a classification algorithm for differentiating patients with MCI from AD patients. The algorithm first uses VBM to normalize the input brain image data and then uses the SVM for the classification process, which tends to ignore potential lesion features due to its overreliance on image preprocessing. Pan et al. [4] designed a multiview and a separable pyramid network, based on deep learning. The network uses depthwise-separable convolution, in order to extract corresponding features from various PET images' slices, thereby preserves as much spatial information as possible and reducing the number of required parameters. This network achieved 83.05% classification accuracy when used to predict patients with MCI. Yee et al. [5] proposed a three dimensional CNN with a residual structure for the AD prediction from 3D PET images; this approach uses batch normalization to normalize the features of each channel and adds instance normalization with a leaky rectified linear unit (ReLU) before each convolutional layer to enhance the generalization and robustness of this model. The AD classification accuracy of the model reaches 81.1%.

The classification accuracy of most AD classification networks is improved by simply adding the layers in the neural network. This practice tends to lose global image information, resulting in poor MCI classification accuracy. At the same time, due to the redundant information, high noise, and severe artefacts in PET images, the lesion features of MCI images cannot be accurately extracted, which further increases the difficulty of accurately distinguishing patients with MCI.

Aiming at the above problems, an AD prediction algorithm based on group convolution and a joint loss function is proposed. The algorithm uses a residual group convolution network as the backbone network, incorporates a hybrid attention mechanism into the backbone network to improve the learning of informative features, and then adds a joint loss function to increase the generalization of this model. We summarize below the new contributions of the paper.

1. ResNet18, based on the group convolutional network, is used as a basic network to complete the action of feature extraction; it uses the same topology to extract lesion features from multiple channels, in order to have an improvement of the network's expression ability
2. A hybrid attention mechanism is introduced after the network's convolutional layer to fully extract the features of the lesion region that makes the network have the function of adaptively learning the feature weights of lesion regions and thus, identify focal regions that are related to disease diagnosis
3. A joint loss function is designed to add a regularization loss function to the traditional cross-entropy loss function to present overfitting and increase the generalization of the model

The rest of the paper is organized as follows: in the related work section, the development achievements and some existing problems in the field of Alzheimer's disease prediction in recent years are introduced, and the innovation points of this paper are demonstrated according to these problems. In the material part, the source of the data set used in this paper and the specific method of preprocessing are introduced. In the method section, we introduce the group convolution, hybrid attention mechanism, and joint loss function in turn in detail. In section “experimental results and analysis”, the experimental settings, evaluation criteria, model visualization, parameter experiment, ablation experiment, and comparison experiment in this paper are elaborated in detail, and the experimental results are analyzed. In the conclusion section, the content of this paper is summarized.

## 2. Related Work

Recently, the great success of CNNs' application in medical image classification has been closely related to the high-speed progress of neural network models. Yang and Liu [6] used AlexNet-5 based on the convolution capable of fast feature embedding for the prediction of the risk of AD prevalence. Jo et al. [7] combined the multilayer basic neural networks with CNNs to extract features from the neuroimaging data. Ding et al. [8] used the neural network based on Inception v3 structure for AD prediction from PET images; this approach uses 11 Inception modules, each consisting of convolutional and pooling layers. However, the practice of simply adding the number of layers can result in the loss of lesion features during convolution, which prevents the accurate identification of patients with MCI. We conceive a neural network structure that can effectively solve this problem, using the same topology for group convolution.

It is generally believed that the study of human vision is the origin of attention mechanism. The brain's information processing capacity is limited, so when facing too much information, humans will selectively give attention to some of it. The rest of the information is ignored. Woo et al. [9] conceived the convolutional block attention module for generating channel and spatial attention feature maps to increase the expressiveness of CNNs. Han et al.'s [10] attention model can extract the features of different regions according to the attributes, so the model is capable to effectively discriminate the content in images, which is considered as an attribute-aware model. Suk and Shen [11] used a variety of SVM to complete the classification. Based on these complex SVM, they built a network prediction model with an automatic encoder to predict advertisements. The attention mechanism has a perfect result in medical image analysis, so we propose adding a hybrid attention model to our neural network to achieve the prediction network focus on more image areas, reduce the attention paid by the network to image redundant information, and enhance network capabilities of learning informative features.

Mikolov et al. [12] proposed the softmax function. For a multiclassification problem, assuming the category label *y* ∈ {1, 2, ⋯, *C*} and given a sample *x*, the softmax function returns the conditional probability that *x* is belonging to category *c*. The softmax function, which uses the cross-entropy loss function to learn the optimal parameter matrix, which may result in overfitting in cases with small samples. Therefore, a regularization operation is required to constrain its parameters to prevent overfitting. Robert [13] and Krogh and Hertz [14] stated *L*_1_ and *L*_2_ regularization, respectively, to limit the growth of weights, reduce the complexity of networks, and thus effectively alleviate the overfitting problem through the *L*_1_ and *L*_2_ paradigms. The dropout operation trains different networks by randomly dropping connections between neurons in each training epoch, eventually fusing all models to predict the output. However, the current mainstream regularization operations constrain the weights of neural networks and do not regularize the output distribution. For PET image classification, the interclass distances between NC patients, patients with MCI, and AD patients are small, and the intraclass distances are not large. The use of mainstream regularization operations has limited the achievable in classification accuracy improvement. We conceive that a joint loss function is added to a regularization loss function to the traditional cross-entropy function, in order to prevent overfitting phenomenon, increase the generalization of the model, and have an improvement on its prediction accuracy.

## 3. Material

### 3.1. Dataset

Data used in preparation of this paper were obtained from the Alzheimer's Disease Neuroimaging Initiative (ADNI) database (http://adni.loni.usc.edu). The ADNI was launched in 2003 as a public-private partnership, led by the Principal Investigator, Michael W. Weiner, M.D.. The primary goal of ADNI has been to test whether serial magnetic resonance imaging (MRI), positron emission tomography (PET), other biological markers, and clinical and neuropsychological assessment can be combined to measure the progression of mild cognitive impairment (MCI) and early Alzheimer's disease (AD). As such, the investigators within the ADNI contributed to the design and implementation of ADNI but did not participate in analysis or writing of this paper.

ADNI-1 and ADNI-2 are two different research phases in the ADNI database. We use 190 AD cases, 350 MCI cases, and 200 NC cases among PET images as the training data from ADNI-1. Four hundred PET images are selected as the test data from ADNI-2. The detailed distributions of the dataset samples are displayed in Table 1.

### 3.2. Data Preprocessing

The PET image data downloaded from the ADNI database are in 3D format. Although the current 3D neural networks have achieved good results in terms of extracting neural image features [15], far more parameters are needed to build a 3D neural network than a 2D network, so more data are required for training to prevent accuracy degradation caused by overfitting. Unlike when addressing natural image datasets, it is still a challenge to collect sufficient medical neuroimaging data, and shape and size differences are present among the different individuals in PET images, so it is difficult to build a high-precision 3D prediction network.

To reduce the data volume of PET images and save computing costs, this paper decomposes the 3D brain PET images into 2D slices for model training. This operation requires a series of preprocessing steps to be conducted on the PET images. The specific process is as follows. First, the 3D PET image data are normalized to an International Brain Mapping Consortium template by the SPM tool [16]. Then, we performed special processing on the images, including averaging, alignment, and interpolation to achieve standard voxels, and their intensities are normalized; the other parameters are set to their default values to obtain images of size 79 × 95 × 79. Finally, each 3D PET image is sliced and tiled into a 2D image sequence using the Python image data preprocessing library. The final image size is 95 × 79. To filter out regions that are not related to classification, such as skulls, the first 10 and last 10 slices images are discarded, and the remaining images slices are used as the dataset in this paper.

## 4. Methods

This chapter elaborates the structures of the network model we conceived and its advantages, including the group convolution module, hybrid attention mechanism, and joint loss function.  Figure 1 presents the AD prediction network structure used in the paper. This network is an improved version of ResNet18. First, the single branch convolution is adjusted to a group convolution of 32 branches, and each convolution branch performs three convolutions. There are two convolution kernels of 1 × 1 size and one convolution kernel of 3 × 3 size. Group convolution increases the width of the network and improves the expressiveness of the model. Then, the feature maps obtained by group convolution are summed up and sequentially went through the channel attention module and spatial attention module, so that the network adaptively learns the importance levels of different features, achieves an enhanced ability to learn informative features from PET images, and suppresses the redundant features. Finally, when all the convolution operations are completed, the obtained feature maps are input in the global average pooling layer, in order to enhance the relationships between features and categories. While preventing model overfitting, it can also improve the robustness and generalization performance of the model because no parameters are required in this layer.

### 4.1. Group Convolution

The current mainstream view is that, adding the depth and width of the network can effectively help us getting a good performance of a CNN. As a classic network, the Visual Geometry Group (VGG) network utilizes stacking blocks to add the depth of the network model, and the deep CNN models proposed afterwards use this strategy as well [17]. However, as the network size increases, the parameters of the network also increase dramatically, which inevitably leads to overfitting when the training data are insufficient, and the large number of parameters leads to a reduced training speed. Therefore, it is difficult to apply the above method to practical engineering problems. Szegedy et al. [18] designed the Inception structure, which extracts features simultaneously and decomposes the sparse matrices into dense matrices, in using various convolution kernels with unequal sizes. Richer features lead to higher accuracy in the final classification results, and areas with more 0 values can no longer be computed, thus greatly reducing the number of required calculations and speeding up the convergence process.  Figure 2 shows a simple split-transform-merge structure. Given D-dimensional input data *x* = [*x*_1_, *x*_2_, ⋯, *x*_*d*_] with input weights *w* = [*w*_1_, *w*_2_, ⋯, *w*_*d*_], a linear activation neuron with no bias is ∑_*i*=1_^*D*^*w*_1_*x*_1_.

However, the different topologies of different branches in the Inception structure require a large number of hyperparameters to be adjusted during the training process and the computational cost will increase significantly [19]. In this research, we conceive an improved Inception structure, group convolution, using the same topology in different branches, as shown in Figure 3. The given PET image is input into a group convolution with 32 branches, and each convolution branch performs three convolutions with one 3 × 3 convolution kernel and two 1 × 1 convolution kernel. Then, the obtained feature maps are additively fused. The use of the same topology increases the network width, enhances the model's generalization, and makes the features learned by the model more diverse.

We combine the group convolution utilizing the same topology with the ResNet18 network to propose the G_ResNet18 network. For PET images, the features in lesion regions are often lost during the convolutional process of a deep convolutional network because of its large amount of redundant information, which makes discriminative lesion features' extraction more difficult. The G_ResNet18 network can extract lesion features from multiple channels to avoid the loss of image features during convolution and improve the accuracy of classification.

### 4.2. Hybrid Attention Mechanism

Taking Conv 1 as a sample, in Figure 4 the feature map *X* ∈ *R*^112×112×64^ obtained by group convolution is used as input. First, both global max pooling (GMP) and global average pooling (GAP) are performed on the input by channel, and the two generated one-dimensional vectors are input in the fully connected layer operation to generate a one-dimensional channel attention *M*_*C*_ ∈ *R*^112×1×1^. Then, multiply the feature map *X* with the channel attention to obtain the channel attention feature map *X*′. Next, GMP and GAP are performed according to the space, and the two two-dimensional vectors generated after pooling are subjected to convolution to obtain a two-dimensional spatial attention *M*_*S*_ ∈ *R*^1×112×64^. Finally, the spatial attention multiplied *X*′, and we can get the attention feature map.

The channel attention mechanism adds attention modules in different channels of the convolutional network. Through self-learning, two fully connected layers are used to acquire the loss of every channel in the feature map. Subsequently, the feature map weights that favour the decreasing loss function according to this loss are made larger. Finally, the feature map is weighted and fused with the original one, in order that the neural network can give more attention on the important feature channels [20].  Figure 5 presents the channel attention module. Firstly, for the feature maps *X* ∈ *R*^112×112×64^, we separately perform a GMP and a GAP on them to acquire two 1 × 1 × 64 feature maps. Then, the obtained feature maps are input into a multilayer perceptron (MLP) consisting of two fully connected layers. After that, the feature maps obtained in the MLP are summed and went through the sigmoid function, so as to obtain weight coefficients between 0 and 1. Finally, the weight coefficients are multiplied by the feature map *X*, and we can acquire the channel attention feature map. The formula for the channel attention mechanism is shown below:

(1) $$\begin{array}{c} M_{c}\left(X\right)=\delta \left(\text{MLP}\left(\text{AvgPool}\left(X\right)\right)+\text{MLP}\left(\text{MaxPool}\left(X\right)\right)\right)=\delta \left(\omega_{1}\left(\omega_{0}\left(X_{\text{avg}}\right)\right)+\omega_{1}\left(\omega_{0}\left(X_{\max}\right)\right)\right), \end{array}$$

where MLP is a multilayer perceptron, AvgPool denotes GAP, MaxPool represents the GMP,  *X* is the feature map, and *δ* is the sigmoid function.

Spatial attention mechanism adds attention modules in the spatial domain of the convolutional network, assigns corresponding importance levels to different positions of the feature map, enhances important regions, and suppresses unimportant regions [21].  Figure 6 reveals the spatial attention module. First, each feature map in *X* ∈ *R*^112×112×64^ is subjected to GMP and also GAP, and then the multichannel features are compressed into a single channel through a 7 × 7 convolution kernel to eliminate the influence of the information distribution between channels. After that, the spatial weight is normalized through a sigmoid function. Finally, the feature map *X* multiply with the weights, so that we can acquire the spatial attention feature map. The formula for the spatial attention mechanism is shown below:

(2) $$\begin{array}{c} M_{s}\left(X\right)=\delta \left(f^{7\times 7}\left[\text{AvgPool}\left(X\right);\text{MaxPool}\left(X\right)\right]\right), \end{array}$$

where AvgPool is the GAP and MLP is the multilayer perceptron, MaxPool is the GMP,  *X* is the feature map, and *δ* is the sigmoid function.

In clinical practice, different individuals have different absorption capacities with respect to the imaging agents, which makes their PET images have certain differences. At the same time, the features of PET images are not obvious, which makes it difficult for a general convolutional network to extract valid features. Therefore, many researchers have chosen to embed modules that have fewer parameters and focus on disease lesion regions into their algorithms when performing disease prediction tasks. To enhance the valid features of PET images and suppress redundant and invalid information, we use a hybrid attention mechanism. The features of the lesion region of PET images are fully extracted using two different attention modules, which strengthen the deep semantic nature of the features, enable the network to adaptively reduce the attention paid to redundant information, and further improve the network's learning ability of informative features.

### 4.3. Joint Loss Function

Cross-entropy loss function is considered to be the most common loss function in the task of image classification, which utilizes the softmax function to obtain the confidence of each category, and then calculates the cross-entropy loss. We defined here the cross-entropy loss function as following:

(3) $$\begin{array}{c} L_{\text{cross}-\text{entropy}}=-\frac{1}{N}\overset{N}{\underset{i=1}{\sum }}\overset{3}{\underset{j=1}{\sum }}\left[y_{i}\ln p_{i,k}\right], \end{array}$$

where *N* is the samples' total number; *y*_*i*_ denotes the labels, which correspond to AD patients, patients with MCI, and NC patients in this paper; and *p*_*i*,*k*_ is the softmax function's output, which indicates the probability that the *i* th sample is one of the *k* th category.

We defined the regularization loss function as following:

(4) $$\begin{array}{c} L_{\text{reg}}=\frac{1}{2}\overset{N}{\underset{i=1}{\sum }}{\left\|\left.f_{i}-C_{y_{i}}\right\|\right.}^{2}, \end{array}$$

where *f*_*i*_ is the *i*th sample's feature vector. The center of the feature class of *y*_*i*_ is *C*_*y*_*i*__, which is updated during each epoch by Equation (5), where *α* is the learning rate and *φ* is the delta function.

(5) $$\begin{array}{c} C_{j}=C_{j}-\alpha {\Delta C}_{j}=C_{j}-\alpha \frac{\partial L_{\text{reg}}}{\partial C_{j}}=C_{j}-\alpha \frac{\sum_{i=1}^{N}\varphi \left(y_{i}==j\right)\left(C_{j}-f_{i}\right)}{1+\sum_{i=1}^{N}\varphi \left(y_{i}==j\right)}. \end{array}$$

Thus, the joint loss function *L* proposed in this paper is defined as

(6) $$\begin{array}{c} L=L_{\text{cross}-\text{entropy}}+{\beta L}_{\text{reg},} \end{array}$$

where *β* is a hyperparameter that regulates the balance between the interclass and intraclass losses. When *β* = 0, it is said that the joint loss function degenerates into the cross-entropy loss function. In this paper, *β* is set to 0.01, and the argumentation process is described in Section 5.4 (Parameter Experiments).

## 5. Experimental Results and Analysis

### 5.1. Experimental Setup

In this paper, experiments are performed in Windows 10, and the algorithm is implemented based on the Python 3.9 and the PyTorch-GPU. The main hardware configurations are introduced in Table 2, and all experimental parameters involved are shown in the next table (Table 3).

### 5.2. Evaluation Indicators

Sensitivity (SEN) is considered to be the probability of correctly diagnosing patients with AD or MCI, and specificity (SPE) refers to the probability of NC patients being correctly diagnosed. We use the following equations to compute the accuracy, sensitivity, and specificity:

(7) $$\begin{array}{c} \text{Accuracy}=\frac{\text{TP}+\text{TN}}{\text{TP}+\text{TN}+\text{FP}+\text{FN}}, \end{array}$$

(8) $$\begin{array}{c} \text{Sensitivity}=\frac{\text{TP}}{\text{TP}+\text{FN}}, \end{array}$$

(9) $$\begin{array}{c} \text{Specificity}=\frac{\text{TN}}{\text{TN}+\text{FP}}, \end{array}$$

where TP means the true positives' number, indicating AD and MCI samples' number that are predicted correctly; FN represents false negatives, which means AD and MCI samples' number are incorrectly predicted as NC; FP signs false positives, indicating the NC samples' number that are wrongly predicted as AD or MCI samples; and TN refers to true negatives, indicating the NC samples' number that are classified correctly.

In practice, the receiver operating characteristic (ROC) curve are often used to compare the predictive performance of various models. The false-positive rate (FPR) is placed on the horizontal coordinate, and the true-positive rates (TPRs) are placed on the vertical coordinates. The formulas of the FPR and TPR are presented as following:

(10) $$\begin{array}{c} \text{TPR}=\frac{\text{TP}}{\text{TP}+\text{FN}}, \end{array}$$

(11) $$\begin{array}{c} \text{FPR}=\frac{\text{FP}}{\text{TN}+\text{FP}}. \end{array}$$

One of the better performances of model B than model A is that the ROC curve of B can completely “wrap” the curve of A. Meanwhile, if that two curves cross, it is difficult to generally conclude which is better. In this case, their areas under the ROC curves (AUCs) should be compared [22]. We make the following assumption that the coordinate connection points together from the ROC curve: {(*x*_1_, *y*_1_), (*x*_2_, *y*_2_), ⋯, (*x*_*m*_, *y*_*m*_)}(*x*_1_ = 0, *x*_*m*_ = 1). The AUC formula is as follows:

(12) $$\begin{array}{c} \text{AUC}=\frac{1}{2}\overset{m-1}{\underset{i=1}{\sum }}\left(x_{i+1}-x_{i}\right)\cdot \left(y_{i}+y_{i+1}\right). \end{array}$$

### 5.3. Model Visualization

To investigate the feature learning process of the proposed AD prediction model, we design a model visualization experiment. The heat map produced during the model training process is shown in Figure 7; that is, the features obtained from the convolution layer through the deconv operation are presented [23]. As seen in Figure 7(a), the model gradually strengthens its focus on the frontal cortex, internal olfactory cortex, hippocampus, and occipital region of each AD sample during the training process. These areas are lesions found in clinical research [24]. As shown in Figure 7(b), the model pays more attention to the superior parietal lobe, middle frontal gyrus and postcentral gyrus of the MCI samples than those of the AD samples. This is in line with clinical studies on MCI [25], indicating that the model we conceived has the capacity of identifying the lesion regions of patients with MCI. As seen in Figure 7(c), the model is more sensitive to the occipital and temporal lobes of the NC samples. Therefore, the regions of interest of the proposed model are consistent with the findings in clinical research and are interpretable.

### 5.4. Parameter Experiments

To evaluate the contribution of the parameter *β*, we design a parametric experiments in which the other conditions are the same and only parameter *β* is different.  Table 4 below introduces the experimental results.

As seen in Table 4, when *β* = 0, the joint loss function degenerates into a cross-entropy loss function, and compared to the best results the prediction accuracy and AUC decrease by 2.1% and 2.3%, respectively. When *β* < 0.01, the prediction accuracy and AUC increase with increasing *β*. When *β* > 0.01, the prediction accuracy and AUC decrease with increasing *β*. At present, it is still difficult to collect enough PET images. When the amount of data is small, the joint loss function regularizes the output distribution, thereby preventing overfitting, increasing the generalization of the model, and improving its prediction accuracy.

### 5.5. Ablation Experiments

To evaluate the contributions of the group convolution and hybrid attention mechanism, we design several control groups for ablation experiments.  Table 5 gives the experimental results, and Figure 8 presents the ROC curves. The control groups are set up as follows.

1. ResNet18 is a CNN model with ResNet18 as the backbone network
2. G_ResNet18 is a CNN model with G_ResNet18 as the backbone network
3. G_ResNet18+CAM is a CNN model that adds a channel attention mechanism to G_ResNet18
4. G_ResNet18+SAM is a CNN model that adds a spatial attention mechanism to G_ResNet18
5. G_ResNet18+HAM is a CNN model that adds a hybrid attention mechanism to G_ResNet18

As seen in Table 5 and Figure 8, compared with those of ResNet18, the classification accuracy of G_ResNet18 using group convolution improves by 13.5%, and the AUC improves by 9.4%. This demonstrates the effectiveness of the group convolutional network for the three classification tasks. G_ResNet18 uses group convolution to prevent the loss of image features during convolution and to raise the diversity of the observed features. Compared with Resnet18, G_ResNet18 can extract more features that are distinguishable and potential lesion information, so it can learn more detailed features from PET images and achieve improved classification accuracy.

As seen in Table 5 and Figure 9, both the addition of the channel attention mechanism and spatial attention mechanism in G_ResNet18 increases the classification accuracy by 1.8% and 2.3%, respectively, and the AUC improves by 1.4% and 2.9%, respectively. The addition of the hybrid attention mechanism in G_ResNet18 improves the classification accuracy by 4.5% and the AUC by 5.3%. The attempt to use the channel attention module and the spatial attention module alone proves that this is not an improvement, but the addition of the hybrid attention mechanism has a greatly improvements on the network's classification results. It is shown that the use of two different attention mechanisms can fully extract the features of lesion regions in PET images, strengthen the deep semantics of these features, enable the network to adaptively reduce the attention paid to redundant information, enhance the network's capacity to learn informative features, and improve the prediction accuracy.

### 5.6. Comparative Experiment

This section compares it with current AD prediction algorithms, and the datasets are all derived from the ADNI database in order to verify whether the algorithm is really effective. The results of the comparative experiments are given in Table 6.

As shown in Table 6, compared with the AD prediction algorithms based on the Inception v3 structure proposed by Ding et al. [8], Sajjad et al. [26], and Lu et al. [27], the algorithm conceived improves the classification accuracy by up to 24%. This shows that the group convolution utilizing the same topology can improve the algorithmic performance, reduce the global information loss, enrich the lesion information extracted by the network, and avoid the errors caused by the singularity of feature extraction. Compared with the AD prediction algorithms based on DensNet proposed by Liu et al. [28] and Solano-Rojas and Villalón-Fonseca [29], the algorithm proposed improves the classification accuracy by up to 21%. This indicates that the hybrid attention mechanism can capture the correlations between features, suppress redundant features, enhance the correlations between features and lesion regions, and perform adaptive feature extraction for regions with more information in PET images, thus further enhancing the recognition capability of the model.

In summary, the algorithm proposed has an effectively improvement in prediction accuracy of patients with MCI.

## 6. Conclusion

It is difficult to accurately predict patients with MCI due to the difficulty of lesion feature extraction and the large amount of redundant information contained in PET images. To address the above problems, an AD prediction algorithm based on group convolution and a joint loss function is proposed. First, a group convolutional backbone network based on ResNet18 is designed to extract lesion features from multiple channels for enhancing the network's expression ability. Then, a hybrid attention mechanism is displayed to fully extract the features of the lesion regions in PET images in order that the network can adaptively give attention to the target regions of learning the feature weights and have enhancement on the network's ability to learn the lesion regions that are relevant to disease diagnosis. Finally, a joint loss function, which puts a regularization loss function into the traditional cross-entropy loss function to prevent overfitting and increase the generalization of the model, is proposed. The research results show that the classification accuracy of the conceived algorithm has a better performance than that of the current mainstream algorithm, which is beneficial to the screening of patients with MCI and thus can achieve AD prediction.

## Figures and Tables

**Figure 1:** (a) is the AD prediction network structure used in this paper; and (b) is the detailed structure of Conv 1.

**Figure 2:** Schematic diagram of the split-transform-merge structure.

**Figure 3:** Group convolution with the same topology.

**Figure 4:** Schematic diagram of the hybrid attention mechanism.

**Figure 5:** Schematic diagram of the channel attention mechanism.

**Figure 6:** Schematic diagram of the spatial attention mechanism.

**Figure 7:** Regions of interest yielded by the proposed model: (a) AD samples, (b) MCI samples, and (c) NC samples.

**Figure 8:** ROC curves produced in the group convolution ablation experiments.

**Figure 9:** ROC curves produced in the hybrid attention mechanism ablation experiments.

**Table 1:** Detailed distributions of samples.

Datasets	Label	Case (n, M/F)	Age (year, mean ± SD)
Train	AD	100/90	75.3 ± 7.5
	MCI	150/100	74.9 ± 7.6
	NC	100/100	75.8 ± 5.0

Test	AD	70/54	74.2 ± 8.0
	MCI	100/92	71.7 ± 7.6
	NC	50/34	74.8 ± 6.8

**Table 2:** Hardware configuration.

Name	Configuration
CPU	Intel i7-12700K@3.6 GHz
GPU	NVIDIA GeForce RTX 3060 12GB
RAM	64GB
Hard drive	1 TB

**Table 3:** Parameter settings.

Parameter	Value
Batch size	32
Number of epochs	100
K_fold	10
Learning rate	0.001
Optimizer	SGD

**Table 4:** Parameter experiment.

Parameter value	ACC (%)	AUC (%)
0	87.5	90.2
0.005	88.9	91.8
0.01	89.4	92.3
0.015	88.6	91.7
0.02	87.9	91.4

**Table 5:** Ablation experiment.

Method	ACC (%)	AUC (%)
ResNet18	75.3	80.1
G_ResNet18	85.5	87.6
G_ResNet18+CAM	87.1	88.9
G_ResNet18+SAM	87.5	90.2
G_ResNet18+HAM	89.4	92.3

**Table 6:** Comparison of the proposed method's results and those of others.

Study	Subjects			Data			Classification result (%)			
	AD	MCI	NC	Modality	Type	Base	SEN	SPE	ACC	AUC
Liu et al., 2017 [28]	121	126	120	2D	PET	ADNI	76.19	70.37	73.82	73.64
Ding et al., 2018 [8]	36	79	73	2D	PET	ADNI	64.67	79	63.67	76.0
Solano-Rojas and Villalón-Fonseca 2021 [29]	95	160	126	2D	PET	ADNI	87.3	83.5	86	—
Sajjad et al., 2021 [26]	30	64	42	2D	PET	ADNI	73	72	72	—
Lu et al., 2020 [27]	238	217	360	2D	PET	ADNI	79.69	83.84	82.93	—
The proposed method	124	192	84	2D	PET	ADNI	87.43	88.26	89.4	92.3

## Data Availability

In this research, the data we used are from ADNI public database, which can be openly downloaded on the website.
